# Effect of lung flooding and high-intensity focused ultrasound on lung tumours: an experimental study in an *ex vivo* human cancer model and simulated *in vivo* tumours in pigs

**DOI:** 10.1186/2047-783X-19-1

**Published:** 2014-01-07

**Authors:** Frank Wolfram, Carsten Boltze, Harald Schubert, Sabine Bischoff, Thomas Günther Lesser

**Affiliations:** 1 Department of Thoracic and Vascular Surgery, SRH Wald-Klinikum Gera, Teaching Hospital of Friedrich-Schiller-University of Jena, Strasse des Friedens 122, D-07548 Gera, Germany; 2 Department of Pathology, SRH Wald-Klinikum Gera, Teaching Hospital of Friedrich-Schiller- University of Jena, Strasse des Friedens 122, D-07548 Gera, Germany; 3 Institute of Animal Experimentation, Friedrich-Schiller University of Jena, Bachstrasse 18, D-07743 Jena, Germany

**Keywords:** High-intensity focused ultrasound, Lung cancer ablation, Lung flooding

## Abstract

**Background:**

High-intensity focused ultrasound is a valuable tool for minimally invasive tumour ablation. However, due to the air content in ventilated lungs, lung tumours have never been treated with high-intensity focused ultrasound. Lung flooding enables efficient lung sonography and tumour imaging in *ex vivo* human and *in vivo* porcine lung cancer models. The current study evaluates the effectiveness of lung flooding and sonography-guided high-intensity focused ultrasound for lung tumour ablation in *ex vivo* human and *in vivo* animal models.

**Methods:**

Lung flooding was performed in four human lung lobes which were resected from non-small cell lung cancers. B-mode imaging and temperature measurements were simultaneously obtained during high-intensity focused ultrasonography of centrally located lung cancers. The tumour was removed immediately following insonation and processed for nicotinamide adenine dinucleotide phosphate-diaphorase and H&E staining. In addition, the left lungs of three pigs were flooded. Purified BSA in glutaraldehyde was injected centrally into the left lower lung lobe to simulate a lung tumour. The ultrasound was focused transthoracically through the flooded lung into the simulated tumour with the guidance of sonography. The temperature of the tumour was simultaneously measured. The vital signs of the animal were monitored during the procedure.

**Results:**

A well-demarcated lesion of coagulation necrosis was produced in four of four human lung tumours. There did not appear to be any damage to the surrounding lung parenchyma. After high-intensity focused ultrasound insonation, the mean temperature increase was 7.5-fold higher in the *ex vivo* human tumour than in the flooded lung tissue (52.1 K ± 8.77 K versus 7.1 K ± 2.5 K). The transthoracic high-intensity focused ultrasound of simulated tumours in the *in vivo* model resulted in a mean peak temperature increase up to 53.7°C (±4.5). All of the animals survived the procedure without haemodynamic complications.

**Conclusions:**

High-intensity focused ultrasound with lung flooding produced a thermal effect in an *ex vivo* human lung carcinoma and *in vivo* simulated lung tumours in a porcine model. High-intensity focused ultrasound is a potential new strategy for treating lung cancer.

## Background

Lung cancer remains the leading cause of cancer-related death in the western population [1,2]. In addition to primary tumours, the lung is the most common site for metastatic spread of other malignancies. Curative treatment of lung tumours or metastases requires surgical resection, which results in the loss of functional lung parenchyma. Unfortunately, fewer than half of patients are eligible for curative surgery due to limited lung function [3]. Radiation or chemotherapy alone rarely cures patients. Minimally invasive local ablation (for example, percutaneous laser or radiofrequency) results in major complications in 6% of patients and procedure-specific 30-day mortality rates of 2.6% [4]. Furthermore, the local progression rate is 35% [5]. Therefore, these procedures are palliative strategies.

High-intensity focused ultrasound (HIFU) is a non-invasive, highly precise procedure to locally destroy tissue through ablation. Current clinical trials are evaluating the effectiveness of HIFU for the treatment of cancers of the brain, breast, liver, bone, and prostate [6-9]. However, lung cancers have never been treated with this approach, because the ventilated lung is a total acoustic absorber and reflector [10]. This problem was solved by lung flooding. Lung flooding enables efficient lung sonography and tumour imaging in *ex vivo* human and *in vivo* porcine lung cancer models [11]. The conditions for applying HIFU to lung tumours are provided.

The aim of this study was to evaluate the effectiveness of sonography-guided HIFU with lung flooding for lung tumour ablation in *ex vivo* human and *in vivo* animal models.

## Methods

### *Ex vivo* examinations

#### Preparation of resected human lung lobes with carcinoma

Four patients with non-small cell lung cancer (NSCLC) received therapeutic lobectomies of the right lower lobe (n = 2), right upper lobe (n = 1), or left lower lobe (n = 1). The average age of the patients was 75.7 years (range 68 to 82 years). The mean tumour diameter was determined by computed tomography and was 4.1 cm (range 3.2 to 5.1 cm). Pre-surgical histological diagnoses of three adenocarcinomas and one large cell neuroendocrine carcinoma were confirmed with percutaneous or transbronchial needle biopsies. The lobes were cooled in a 15°C isotonic liquid bath immediately following resection and prepared for liquid filling (flooding) *in tabula*. An expanded polytetrafluoroethylene graft was then anastomosed end-to-end with the lobar bronchi. An infusion system was connected to the conduit, and the lobes were continuously filled with isotonic saline (15°C) until the functional residual capacity was reached. The lung lobe was examined transpleurally by ultrasound (MicroMaxx™ Portable Ultrasound System; SonoSite, Inc., Bothell, WA, USA) in the liquid bath with a linear probe (L38e, 10 to 5 MHz; SonoSite, Inc., Bothell, WA, USA) in fundamental B-mode. The lobes were selected for HIFU only in cases with gas-free filling and complete sonographic imaging of the tumour. This study was approved by the ethics committee of the Medical Association of Thuringia.

#### HIFU application

The experimental HIFU setup contained the HIFU transducer H102 (Sonic Concepts Inc., Bothell, WA, USA), a power amplifier (RF Source, Athena, Greece), a Type K thermocouple (XF339, Labfacility Ltd., Sheffield, South Yorkshire, UK), and a digital multimeter (34401A, Agilent, Santa Clara, CA, USA). The HIFU setup and alignment with the tumour are illustrated in Figure 1. The thermocouple was guided through the centre hole of the HIFU transducer into the tumour. The alignment of the HIFU focal zone within the tumour and the thermocouple was monitored by ultrasound with a curved imaging probe (C11e, SonoSite, Inc., Bothell, WA, USA), which was mounted sideways on the HIFU transducer. Self-heating of the thermocouple was excluded by applying HIFU to the thermocouple in water. An impedance-matching network provided by the manufacturer drives the HIFU probe with a radiofrequency (RF) amplifier. The acoustic power of the focal zone in water was estimated to be 2,500 W/cm^2^ at 1.1 MHz (I_SPTP_, spatial peak, temporal peak) based on the manufacturer’s calibration sheet. A duty cycle of 50% and a repetition frequency of 10 KHz were applied. The cancer tissue was exposed to HIFU for ten seconds. The focal zone was immediately moved through the tumour in lateral 2 mm increments. HIFU was initiated again for ten seconds, and ultrasound B-mode imaging was then performed. HIFU exposure ended after one slice of the HIFU zone moved through the tumour volume. Subsequently, the HIFU focus and thermocouple were placed into flooded lung tissue. The procedure was repeated as described above. All experimental steps were performed within 45 minutes of surgical resection.

**Figure 1:** **Schematic setup of *ex vivo *high-intensity focused ultrasound application.** High-intensity focused ultrasound transducer (1), flooded lung (2), cancer (3), attenuator (4), impedance matching network (5), power RF amplifier (6), signal generator (7), thermocouple (8), multimeter (9), thermo-control (10), and sector-array probe (11).

#### Histopathology and enzyme histochemistry

The specimen, including the tumour, was cut at a 90° angle to the treated cross section immediately following the last HIFU exposure. Each half of the tumour was sectioned parallel to the cutting surface to show the transition from ablated to non-ablated tumour. One part was fixed in 4% formaldehyde for H&E, and the other was frozen in liquid nitrogen for nicotinamide adenine dinucleotide phosphate (NADPH)-diaphorase staining. An intralobar metastasis from one case served as an untreated tissue control.

### *In vivo* examination

#### Animal preparation

Animal experiments were performed on three female pigs (Deutsches Landschwein breed; weight range: 33 to 38 kg, average: 35.5 kg) with permission from the Veterinary Department of the Thuringian State Authority for Food Protection and Fair Trading in compliance with the National Animal Protection Act. Total intravenous anaesthesia was initiated with propofol (10 mg/kg/h), fentanyl (0.05 to 0.08 μg/kg/min), and pancuronium bromide (2.5 μg/kg/min). A left-sided Robertshaw double-lumen tube with an extra-long bronchial lane (size 39 Ch; special product by Mallinckrodt Medical, Dublin, Ireland) was inserted after tracheotomy. Mechanical ventilation was performed with an ICU respirator (Servo 900, Siemens AG, Munich, Germany) on a volume-controlled setting (FIO_2_ = 1.0; tidal volume 10 ml/kg; respiratory rate 16 to 20/min; positive end expiratory pressure = 6 cm H_2_O). The electrocardiogram, arterial blood pressure, capillary oxygen saturation, and expiratory CO_2_ concentration were measured and recorded continuously (Datex AS/3 Compact Multiparameter Patient Monitor; Datex-Ohmeda Corp., Helsinki, Finland). Arterial blood gases were analysed every 30 minutes (ABL System 625; Radiometer Medical, Copenhagen, Denmark).

#### Tumour simulation and HIFU application

The HIFU setup for transthoracic application on pigs contained a self-manufactured sample holder. The HIFU transducer (SU102, Sonic Concepts Inc., Bothell, WA, USA) was arranged with the sideways attached puncture channel to guide the thermocouple and curved imaging probe (C11e, MicroMaxx; SonoSite Inc., Bothell, WA, USA). The three elements were arranged such that the thermocouple tip was in the focus of the HIFU beam. A rib was resected after lung flooding without pleural injuries. The HIFU applicator was placed above the resected rib (Figure 2). A 17-G needle was placed in the centre of the lower left lung lobe with the guidance of a percutaneous transpleural ultrasound. Five millilitres of a fluid composed of purified BSA and glutaraldehyde (Bioglue®; CryoLife Europa, Guildford, UK) were injected to simulate a lung tumour. A thermocouple was immediately inserted through the needle into the simulated tumour. The alignment of the focal zone with the target lesion and thermocouple was monitored by ultrasound imaging. The surgical HIFU probe with an outer diameter of 35 mm operates at 3.0 MHz. The focal acoustic intensity was estimated to be 2,000 W/cm^2^ MHz (I_SPTP_ , spatial peak, temporal peak) based on the manufacturer’s calibration sheet. HIFU was applied according to a ‘one second on, one second off’ scheme. The temperature inside the simulated tumour was recorded by the thermocouple during HIFU exposure. Data were transferred and stored on a laptop.

**Figure 2:** ***In vivo *high-intensity focused ultrasound application after rib resection.** Thermocouple (1), high-intensity focused ultrasound transducer (2), and sector-array probe (C11e, 8 to 5 MHz, Micromaxx, Sonosite Inc., Bothell, WA, USA) (3).

## Results

### *Ex vivo* examinations

The mean temperature in the tumour tissue increased by 52.1 K ± 8.77 K after ten seconds of HIFU exposure. The same acoustic intensity produced a mean temperature increase of 7.1 K ± 2.5 K in a flooded lung. The temperature increase in the *ex vivo* human NSCLC was 7.5-fold higher than that in the flooded lung tissue (Figure 3). The sonoablated cancer tissue appeared to be strongly hyperechoic immediately following HIFU application (Figure 4). The strength of echogenicity decreased 30 seconds after HIFU exposure but did not disappear. The ablated cancer tissue appeared to be slightly whitish in all four cases. A demarcation between treated and non-treated areas was observed (Figure 5).

**Figure 3:** **Mean temperature increase.** The mean temperature increases (± standard deviation) within an adenocarcinoma surrounded with flooded lung tissue (n = 3) and within flooded lung alone (n = 3) are shown. Temperatures were measured with a thermocouple ten seconds after *ex vivo* high-intensity focused ultrasound insonation.

**Figure 4:** **Sonomorphology of adenocarcinoma in *ex vivo *flooded human lung before and after high-intensity focused ultrasound. (A)** B-mode ultrasound image of adenocarcinoma in flooded lung before *ex vivo* high-intensity focused ultrasound insonation. Adenocarcinoma (1), flooded lung (2), thermocouple (3), and focal zone of high-intensity focused ultrasound beam (4); **(B)** B-mode ultrasound image after single high-intensity focused ultrasound insonation demonstrates a sharply demarcated and strongly hyperechoic sonolesion within the tumour.

**Figure 5:** **Macroscopic appearance of the zone of ablated tumour tissue (inside the highlighted circle) in the resected specimen.** Arrows show the tumour margin of non-ablated adenocarcinoma.

H&E staining showed coagulative necrosis with cytoplasmic eosinophilia, disruption of cellular membranes with blurred cytoplasmic borders, karyolysis, and nuclear pyknosis. Insonated and non-insonated cancer tissues showed sharp demarcations. There was a small region between the area of coagulation necrosis and vital cancer tissue in which cells showed cytoplasmic vacuolization (Figure 6). These characteristics were not found in the untreated areas of cancer tissue. NADPH-diaphorase staining produced a sharp demarcation between ablated and non-ablated cancer tissue, and demonstrated that vital lung tissue was present immediately adjacent to ablated cancer tissue (Figure 7). HIFU-treated tumour tissue did not show evidence of vitality by NADPH-diaphorase staining. Sonographic lesions were not detected in the tumour surrounding the lung tissue or in the direction of the HIFU irradiation. In contrast, a non-treated metastatic tumour in the same lobe showed complete vitality.

**Figure 6:** **Histological examination of large cell neuroendocrine carcinoma immediately after *ex vivo *high-intensity focused ultrasound application.** The border between ablated and non-ablated tumour is shown. There is a vital tumour in the upper left image **(A)**. The thermal effect is visible as a small area, which contains cells with cytoplasmic vacuolization **(B)** and as a coagulative necrosis with cytoplasmic eosinophilia, disruption of cellular membranes with blurred cytoplasmic borders, karyolysis, and nuclear pyknosis **(C)**. Arrows indicate the sonolesion boundary (H&E).

**Figure 7:** **Nicotinamide adenine dinucleotide phosphate (NADPH)-diaphorase staining.** There is a sharp demarcation between vital lung tissue **(A)** and ablated tumour tissue **(B)**. Immediately after *ex vivo* high-intensity focused ultrasound application, NADPH-diaphorase staining showed a lack of uptake of the vitality stain in finger-shaped tumour extensions **(B)**.

### *In vivo* examination

A lung tumour could be simulated in the flooded lung of each of the three animals by sonography-guided injection of BioGlue®. The central tumour appeared hypoechoic by B-mode sonography and was sharply demarcated from the lung parenchyma with small inclusions of air. A temperature rise was monitored within each one-second application of HIFU irradiation. A section of 25 seconds of HIFU exposure in the ‘one second on, one second off’ scheme is shown in Figure 8. Repeated HIFU insonation caused an overall average temperature increase of up to 53.7°C (±4.5, n = 3).

**Figure 8:** **Temperature profile inside the simulated target lesion (BioGlue®).** The temperature profile is shown for the simulated lesion during transthoracic high-intensity focused ultrasound insonation after *in vivo* flooding of the left lung of a pig*.* Temperature increases were monitored for each one-second treatment with HIFU irradiation. A section of 25 seconds of HIFU exposure following the ‘one second on/off’ scheme is demonstrated. The repeated HIFU insonation caused a temperature increase up to 54°C.

Arterial blood pressure, oxygen, and carbon dioxide partial pressure were normal in all three animals during and after HIFU insonation. No animals died during the procedure.

## Discussion

Currently, the best curative treatment for early-stage non-small cell lung cancer and lung metastases is surgical resection. However, surgery is not appropriate for patients with reduced pulmonary function due to the loss of lung parenchyma. Minimally invasive technologies for local tumour control have been developed as alternatives to surgery. The most common method is percutaneous radiofrequency ablation. However, this kind of thermal ablation is limited because the extent to which tissue has been successfully ablated cannot be accurately assessed. This could be a reason for the observed rate of local recurrence. Another risk factor for local tumour progression is the adherence of viable tumour tissue to needle applicators and subsequent spreading of tumour cells [12]. In addition, pulmonary percutaneous radiofrequency ablation is invasive and associated with major complications and mortality.

HIFU has been examined in animal experiments and clinical trials as a technique for localized tissue ablation for more than 60 years. HIFU is superior to other radiation beams, because it penetrates deep and selectively destroys tumour tissue. In addition, HIFU can be applied as many times as needed [13]. HIFU is currently used as a therapy for cancers of the abdominal organs, breast, and brain [14-18].

Non-invasive local therapies with curative intention are not available for lung tumours. HIFU has never been applied to lung tumours, because the air content in ventilated lungs reflects acoustic intensities. We solved this problem with lung flooding. Lung flooding enables efficient lung sonography and tumour imaging in *ex vivo* human and *in vivo* porcine lung cancer models [11]. The cancerous tissue was visualized by replacing the alveolar gas with fluid, facilitating ultrasound-guided HIFU. The aim of the present study was to explore the ability of therapeutic ultrasound to penetrate the overlying lung parenchyma without damage and to increase the temperature of the tumour tissue.

A tissue temperature greater than 60°C will usually cause instantaneous and irreversible cell death within one second in most extrapulmonary tissues due to coagulation necrosis. Coagulation necrosis is the primary mechanism by which HIFU destroys tumour cells [6]. Our *ex vivo* studies showed that lung cancer tissue absorbed acoustic energy, leading to an increase in tumour temperature of 52.1 K. Based on the temperature of a cooled lung lobe (15°C), a peak temperature of 67°C was created. The heat induced by HIFU was sufficient to generate coagulation necrosis in the lung cancer tissue. In contrast, the same acoustic HIFU energy caused a minimal temperature increase (7.1 K) in flooded parenchyma. NADPH-diaphorase staining showed that HIFU was highly selective for tumour tissue in flooded lungs. The lung parenchyma directly adjacent to the ablated cancer tissue was undamaged and viable. This can be explained by the very low attenuation of saline, which is the major mass component in flooded lungs [19]. Thus, the risk of damaging the surrounding tissue or adjacent organs can be minimised as previously described in a study of HIFU in abdominal tumours [20]. A normal saline solution was injected into the abdominal cavity to reduce complications from HIFU therapy for abdominal tumours. This method does not have adverse effects on the efficacy of HIFU ablation [21].

*In vivo* transthoracic HIFU application in pigs caused a mean peak temperature increase up to 53.7°C in a simulated lesion (BioGlue®) deep inside the flooded lung. HIFU energy penetrated through the pleura and flooded lung into the target lesion. The simulated lesion, which was located at a 6 cm depth below the transducer, was heated by HIFU. The temperature increase was highly variable and inconstant. The mechanism of heat generation in the BioGlue®-simulated lesion was unclear. The lesion consisted of purified BSA and glutaraldehyde. Although this simulated lesion was not a true human tumour, the acoustic and thermal properties are similar to those of human cancerous tissue due to similar densities and high protein contents. In addition, movements of the heart and mediastinum may be transmitted to the target lesion, bringing them out of the focal zone.

Lung flooding seems to be ideal for HIFU application, because sonographic imaging is possible and because of other advantages.

Compared to other human tissues, a flooded lung has an ideally suitable beam path, because water has a very low attenuation. In contrast to flooded lung tissue, tumour tissue converts acoustic energy into a therapeutic thermal dose and enables selective heating of the cancer mass. Consequently, damage to healthy lung tissue is minimised.

In addition to acoustic advantages, there are other favourable conditions for tumour ablation in a flooded lung. There is no pulmonary blood flow in a flooded lung [22]. Perfusion reduces heat and is not desirable with locoregional thermal therapy. In addition, ischaemia-related acidosis sensitises tumour tissue to heat. In comparison to a ventilated lung, lung flooding reduces tumour movements caused by breathing.

The following limitations existed in the current study.

The risk of lung flooding in patients with limited lung function is unclear. Further studies on patients with limited lung function should be performed to examine the influence of unilateral lung flooding on haemodynamics and gas exchange. Ongoing studies in pigs showed that lung flooding of only one lobe is feasible.

Transcutaneous application was not applied for the *in vivo* or *ex vivo* studies. One rib had to be resected to apply the HIFU applicator, which consisted of a HIFU transducer and sector-array probe, to the chest of a pig. Technical improvements in the application system are necessary to ensure that the HIFU focal zone is aimed precisely at the target lesion with the guidance of sonography. Transthoracic HIFU application is difficult despite resection of the ribs, because the intercostal spaces in the animal model are narrow. A method and transducers have been developed to avoid the shielding of therapeutic ultrasound by the human rib cage [23].

Different HIFU exposure schemas (ten seconds *ex vivo* versus ‘one second on/off’ *in vivo*) and transducers were applied during this study. Ultrasound imaging is disturbed if HIFU is continuously on. Therefore, the intermittent ‘one second on/off’ *in vivo* schema was needed to control the focal alignment with the thermocouple during the ‘one second off’ interval.

For HIFU application to human tumours, resected lung lobes were used.

The gas-free filling occurs at 71.4% of the resected lobes. This limitation is due to residual air in non-collapsed bronchi that can only solved by resorption under *in vivo* conditions [11]. Lung flooding was performed with cooled saline at 15°C for the *ex vivo* HIFU application to ensure that hypoxic damage did not occur within the tumour and lung tissues. This was important, because the NADPH-diaphorase staining method is based on mitochondrial vitality, which is very sensitive to ischaemia.

A hyperechoic area was found within the tumour tissue immediately following HIFU exposure. Grayscale changes have been shown to be a useful marker for HIFU-induced tissue destruction [8]. However, it is unclear whether the area of grayscale changes corresponds with the ablated area, such that a hyperechoic sonolesion represents irreversibly damaged tissue. B-mode ultrasound imaging is probably not the best method for monitoring tissue response. Currently, the most important problem associated with ultrasound-guided HIFU ablation is the lack of reliable thermometry and lesion production monitoring [6]. In addition to ultrasound imaging, real-time magnetic resonance thermometry could be important for ascertaining the extent of tumour destruction [24-26].

## Conclusions

In combination with lung flooding, high-intensity focused ultrasound produced a thermal effect in an *ex vivo* model of human lung carcinoma and in simulated lung tumours in an *in vivo* porcine model. High-intensity focused ultrasound is a potential strategy for treating lung cancer. Further studies will examine HIFU therapy in animal models of lung cancer.

## Abbreviations

BSA: Bovine serum albumin; FIO2: Fraction of inspired oxygen; HIFU: High-intensity focused ultrasound; H&E: Hematoxylin and eosin; NSCLC: Non-small cell lung cancer; NADPH-diaphorase: Nicotinamide adenine dinucleotide phosphate-diaphorase.

## Competing interests

The authors declare that they have no financial or non-financial competing interests.

## Authors’ contributions

FW was responsible for HIFU technique and temperature measurement. He collected and evaluated the data and wrote the manuscript. HS and SB performed the anaesthesia. CB performed the histopathological and enzyme histochemistry examinations. TGL co-wrote and revised the manuscript and discussed the results with the authors. All authors read and approved the manuscript.
